# Biomechanical Analysis of the Human Knee Joint

**DOI:** 10.1155/2022/9365362

**Published:** 2022-03-04

**Authors:** Sheng Wang

**Affiliations:** Shanxi University, Taiyuan 030006, China

## Abstract

Exercise is an indispensable part of human daily life. The knee joint is inseparable from human movement. The knee is relatively fragile and easy to get injuries. Therefore, the biomechanical properties of knee joints were studied. The VICON T40S 3D motion acquisition and analysis system and the AMTI 3D force measurement platform were used to collect the lower limb kinematics and dynamics data of five male volunteers. Then the knee angle and moment of the human body are analyzed, the foot pressure was obtained by force plate, and the ground reaction force was obtained. The results show that: (1) in terms of knee flexion and extension torques, the peak stretching torques occurred in about 25% and 65% of the gait cycles. At the beginning of the gait, which is the flexion moment, the knee joint produces a moment of −24.65 Nmm, 25% of gait cycles reached the maximum peak value of 896.89 Nmm, 65% of gait cycles reached the second peak value of 315.81 Nmm; (2) The change of reaction force in a gait cycle is: when the ground starts to react, the ground reaction reaches 600 N. At normal times, the ground reaction force rapidly rises to the maximum value of 890 N; when the gait is in the middle of a single support phase, the ground reaction force is 462 N; when the ankle joint moves in plantar flexion, the ground reaction force increases to 830 N again; finally, when the toe is lifted off the ground, the ground reaction force quickly drops to zero; (3) in the course of a gait cycle, the spatial and temporal parameter curve distribution of the subjects was consistent, and the difference was not significant (*P* > 0.05).

## 1. Introduction

The knee joint is the main joint of the human lower limbs. It has a lot of weight-bearing and a large amount of exercise, and it is the hub of lower limb activities. The structure and function of the knee joint are the most complex joints in the human body. Due to the anatomical complexity of the knee joint (three-component bones: femur, tibia, and patella and their surface cartilage tissue; major ligaments: anterior and posterior cruciate ligaments, medial and lateral collateral ligaments, patellar ligaments, meniscus, attached muscle groups, etc.), kinematic complexity (multiaxis three-dimensional motion) and mechanical complexity (pressure, tensile stress, and shear force are simultaneously applied to the knee during motion and these forces vary dramatically with the gait cycle stage), it is of great theoretical significance to study the mechanical system of knee joint. In the sports population, the improper movement mode often causes knee joint injury, for example, the anterior cruciate ligament, the meniscus, and other related structures are damaged. Among them, anterior cruciate ligament injury is a kind of common potential injury, and it often appears as a kind of noncontact injury in sports, such as landing, changing direction, twisting, and other movements.

Research on knee biomechanics mainly includes the influence of movement, joint contact, and soft tissue deformation and force on joint movement and force. Many scholars have studied this issue. The AMTI 3D three-dimensional force platform is equipped with several piezoresistive sensors to measure the pressure changes in different parts of the entire platform, and the changes in force and torque on the *X*, *Y*, and *Z* axes are calculated. Products are widely used in sports science, clinical medicine, ergonomics, military scientific research, aerospace, and other fields. Therefore, the VICON T40S motion capture system and the AMTI 3D force measurement platform are used to collect the kinematic and dynamic data of the lower limbs. Then, the human knee angle and moment values in the human gait cycle are analyzed, and the foot pressure is obtained by using the force plate. The ground reaction force was obtained to analyze the biomechanical properties of the knee joint.

Therefore, the development of new therapies is critical to prevent permanent adaptive changes in posture in patients with knee injuries [1]. Biomechanics: knowledge of biomechanics helps predict stresses in different parts of the knee during daily activities. Biomechanical parameters such as contact pressure, contact area, and maximum compressive stress of the fully extended knee during the gait cycle were evaluated [2].

Understanding the complex biomechanical behavior of injured knee joints is critical in a variety of clinical situations [3]. Chen conducted a biomechanical analysis of the knee joint during take-off and landing [4]. Kumbhalkar et al. conducted a biomechanical study on knee replacement [5]. Chang et al. analyzed the biomechanical properties of ankle cartilage and ligament in BKTS, a typical Tai Chi movement [6]. Zhang et al. used finite element analysis to study biomechanical changes in load distribution of longitudinal tear of the knee joint semilunar angle [7]. Tarnita et al. applied finite element analysis (FEA) to a virtual component consisting of an orthotic device and an osteoarthritic knee joint (OAK) using Ansys Workbench 14.5 software, to study the influence of orthopedic devices on the maximum stress value of knee cartilage [8]. Yong-Jun et al. established the finite element model of the discoid meniscus of the knee by fusing CT and MRI data to provide a reliable finite element model for the study of the discoid meniscus [9]. Abidin et al. analyzed the biomechanical effects of different fixators (cross nail technique) on knee stability after ACL-R. Finite element analysis was performed on the knee joint with a DST graft and fixator [10].

The triangular partial grid model and the tetrahedral element solid grid model of the knee joint are established in this paper. The structure of each part of the model is clear and smooth, the grid continuity is good, and the size is right. The mesh is in line with the actual situation. The quality of the mesh is excellent after several times of optimization, and it can be applied to the relevant finite element analysis well.

## 2. Research Methods

### 2.1. Experimental Scheme Design

In order to obtain the changes in knee angle, force, and moment during a single gait cycle in healthy subjects, VICON T40S 3D motion acquisition and analysis system was adopted in this experiment. The system has a high sampling rate and good real-time performance, with a maximum of 16 million pixels and the fastest capture speed of 120 fps. The instrument is widely used in VR, biological motion mechanics, human engineering research, physical education, robot design, and other research fields.

The experimental equipment used 10 cameras with a frequency of 100 Hz and sensors with light-emitting spheres, making it easy for the camera to pick it up. In addition, three three-dimensional force measuring plates with an acquisition frequency of 1500 Hz, a T-type calibration frame, and computer and data transmission-related equipment was added. The 3D force plate and the motion capture system are connected with the computer software to collect the gait data needed for the experiment at the same time. Finally, VICON Nexus, a data processing device, corrected the data and calculated the data.

The experiment involved five men, all healthy and able to walk naturally. The lower limbs were normal, and there was no history of knee joint problems. The specific operation is in the shooting area of the laboratory staff around the T-shaped correction frame. The method is to obtain the camera position by collecting the marker movement data. After the calibration begins, the camera continuously collects the data of the marker point, and the marker light on the camera can show the collection situation of the camera. When the blue indicator blinks until the green indicator turns on, the camera has collected enough data. When all 10 cameras complete the collection, the system will automatically stop the collection and start calibration calculation. Successful calibration for each camera is to collect more than 1000 frames of effective data.

In the experiment, each subject was required to add 26 marker points as shown in Figure 1, head (RFHD, LFHD, LBHD, and RBHD), torso (CLAV, C7, RBAK, and T10), points of the pelvis (LASI, LPSI, RASI, and RPSI), lower limbs (RANK, RWRB, RTHI, RKNE, RTIB, LANK, LTIB, LKNE, LTHI, and LWRB), and toes (RTOE, LTOE, LHEE, and RHEE). The points captured by the camera are synthesized by the computer to obtain the kinematic indexes.

### 2.2. Experimental Data Collection

In order to reduce the influence of various factors on the human body while walking, before the experiment, subjects were asked to do a small amount of walking on their own in the most relaxed state along the route beforehand, familiarize themselves with the route, and experiment when they are not nervous. The experiment process is as follows: first, the basic information of the subject is filled and the measurement data by manual measurement in the computer system; second, the subjects should establish a static model, with their arms spread in a T-shape and their feet spread about 20 cm, in standard standing posture, stand with toes facing forward on the force plate, and hold still. After the markers were identified by VICON, the skeleton model of the subject was established. All subsequent experiments were performed under this model. The line where the flat force plate is located is the route for the subjects to walk. Finally, each participant was asked to walk at a natural walking speed on a set path, ensuring that the force plate had a full gait cycle. There is a five-minute break between each walk so as to not cause fatigue and affect the final results. One subject is required to complete 15 sets of valid data test experiments to ensure that the data has more than 10 sets of optional data. Finally, the data of each cycle of walking in the same direction were extracted from the 15 groups of data.

## 3. Results Analysis and Discussion

The VICON motion capture system defines the angle of the knee joint as follows: the reference line is the extension line of the long axis of the femur, the angle is between the reference line and the long axis of the tibia; knee flexion, adduction, and internal rotation were positive, while the opposite movement was negative; the simulated spatial cartesian coordinate system in the VICON motion capture system defines the *X*, *Y*, and *Z*-axis coordinates of the marked points, where the *X*-axis coordinates are defined as the left and right directions of the spatial origin, the *Y*-axis coordinates are defined as the front and back directions of the spatial origin, and the *Z*-axis coordinates are defined as the upper and lower directions of the spatial origin. Since the knee joint is mainly in the sagittal plane during walking, that is, the *Y*-axis in the VICON system, the kinematics of this study mainly focus on the movement on the *Y*-axis.

In order to process the large amount of data obtained in the experiment, the data required in this experiment can be extracted by using Mokka software, Mokka software can directly visualize data information, as shown in Figure 2. The import format is C3d, and the data collected by gait is imported into Mokka, the first and second landing moments of the left and right heels are respectively treated as a gait cycle. Finally, the knee joint angle value, the plantar pressure value on the force plate, the motion trajectory of the marked point on the *Y*-axis, and the three azimuth torque component values on the knee joint can be extracted and selected during preservation. The observation method of time selection is to intercept a complete gait cycle on the time axis and the data is exported in Excel format.

As shown in Figures 3 and 4, a 27-year-old subject with a weight of 75 kg and a height of 180 cm was taken as an example. The standard deviation of 15 groups of data of knee joint angle and moment was obtained by average processing, and the movement of the knee joint was analyzed accordingly. In the Figures 3(a)–3(d) are the angles and torques of the left and right knee joints, respectively, the solid line of each figure is the average value of the 15 groups of experimental data, and the gray band is the error band.

We select 1, 5, and 10 kinds of materials for the femur model, respectively, and assign values to the femoral materials by the uniform method. That is, we subdivide the gray value of the femoral body mesh into 1, 5, and 10 parts, and each small interval represents an each small area, which is represented by a central gray value, and each material is represented by a different color. Then we determine the expression of the femur, the expression of elastic modulus, and the Poisson's ratio to set the parameters of the material according to the relevant reference books and the referenced literature is

(1) $$\begin{array}{c} \text{Density}=-13.4+1017\times \text{Grayvalue},\\ E-\text{Modu}\times \text{lus}=-388.8+5925\times \text{Density,}\\ \text{Poisson Coefficient}=0.3. \end{array}$$

The time parameters of gait include support time, swing time, and a complete gait cycle time, in which the single support time on one side is consistent with the swing time on the other side. The complete gait cycle time was compared and analyzed. The left leg gait cycle time refers to the time from when the left foot hits the ground until the left foot hits the ground again, and the left foot single support time refers to the time from when the right foot leaves the ground until the right foot hits the ground again; the same is true for the right side. The range of knee joint changes in adolescent gait is affected by many factors. The magnitude of the change in the knee joint becomes smaller and smaller as the grade increases.

It can be seen that the knee angle changes throughout the gait cycle as follows: the knee angle of the left and right legs is about −5° before bending the knee, and the knee angle reaches about 30° when the heel is off the ground at the beginning. During the first landing in the state of bending the knee, the full extension of the knee joint is close to 0°, during the next swing when the gait cycle is about 78% of the complete gait, the knee flexion angle reaches a peak of about 60°, and the next cycle is the foot following the ground. At this point, the knee angle returns to the minimum, as shown in Table 1. However, in the same gait cycle of the left leg and the right leg, the stride length of the left leg is smaller, and the angle difference between the left and right legs is smaller. As can be seen from the figure, the joint angle of the left knee has a slight overextension phenomenon, which is due to the error caused by the inaccuracy between the position of the knee joint sticking point and the standard model.

In terms of knee flexion and extension moments, the peak stretching moments occurred at about 25% and 65% of the gait cycle. At the beginning of the gait, is the flexion moment, the knee produces a moment of −24.65 Nmm 25% of the gait cycle reaches the maximum peak value of 896.89 Nmm, 65% of gait cycles reached the second peak of 315.81 Nmm (see Table 2 for details). The comparison of the initial torque of the gait cycle and the two large peaks of the torque is shown in Figure 5.

In the sagittal plane, the ground reaction curve shows two peaks in a gait cycle. In the early stage of walking, the ground reaction force fluctuates in a small range, and the ground reaction force reaches 600 N after the initial stage of walking. At normal times, the ground reaction force rapidly rises to the maximum value and reaches the maximum value of 890 N. At this time, the ratio of weight to body weight on one limb is 11.8, which is at 20% of the gait cycle. When the gait is in the middle of the single support phase, the value of the force decreases gradually. The curve trough occurs at about 50% of the gait cycle, and the ground reaction force is 462 N. The ratio of this value to the subject's body weight is 6.16. When the ankle is plantar flexion, the ground reaction increases again to a second crest. At this point, it reaches 830 N, which is about 80% of the gait cycle. The ratio of this value to the bodyweight of the walker is 11. Finally, when the toe is off the ground, the ground reaction force quickly drops to zero, as shown in Figure 4. The specific values are shown in Table 3.

In order to verify the validity of the data from this gait experiment, since height also has an impact on the space-time parameters of gait, the left knee joint angles of the subjects aged 22–27 years, average height (175 ± 5) cm, weight (70 ± 5) kg were averaged, and the standard deviation was obtained, as shown in Figure 6. It can be seen from the results that the spatial and temporal parameter curve distribution of the three subjects in a gait cycle is consistent, and there is no significant difference (*P* > 0.05). Therefore, the results can represent the normal gait pattern.

## 4. Conclusions

In terms of the present stage, the curative effect of knee joint replacement surgery, may well solve the patients' pain and basic activities in the short term, but after all, the service life of the knee joint prosthesis is limited, postoperative prosthesis and joint wear, the wear and tear of implants and prostheses remains, so the need to do as much as possible to design a perfect prosthesis. The results showed that: (1) at the beginning of the gait, is the flexion moment, and the knee produces a moment of −24.65 Nmm, 25% of the gait cycle reaches the maximum peak value of 896.89 Nmm, and 65% of the gait cycle reaches the second peak value of 315.81 Nmm. (2) When the gait is in the middle of single support phase, the ground reaction force is 462 N; when the ankle joint moves in plantar flexion, the ground reaction force increases to 830 N again. Finally, when the toe is off the ground, the ground reaction force quickly drops to zero. (3) In the course of a gait cycle, the spatial and temporal parameter curve distribution of the subjects was consistent, and the difference was not significant (*P* > 0.05).

## Figures and Tables

**Figure 1:** Schematic diagram of human test standard points.

**Figure 2:** Importing data in Mokka.

**Figure 3:** Knee angle and moment.

**Figure 4:** Ground reaction force.

**Figure 5:** Initial torque and 2 peak torque of a gait cycle.

**Figure 6:** Verification of the validity of gait data.

**Table 1:** Knee angle changes in a gait cycle.

The gait	Bend your knees before	Heel off the ground	First landing	The second time off the ground	Second landing
The angle(°)	−5	30	0	60	−5

**Table 2:** Peak torque of a gait cycle.

The gait cycle	25%	65%
Peak(Nmm)	896.89	315.81

**Table 3:** Ground reaction force in a gait cycle.

The gait	Feet on the ground (N)	Foot flat (N)	Single supported phase metaphase (N)	Plantar flexion movement (N)	Toe off the ground (N)
Ground reaction	600	890	462	830	0

## Data Availability

The datasets used and/or analyzed during the present study are available from the corresponding author upon reasonable request.
